The article "Effect of Chinese Medicine on the Biological Behavior and Magnetic Resonance Imaging of Bladder Cancer" was published in 2021. Journal: Evid Based Complement Alternat Med.

# Effect of Chinese Medicine on the Biological Behavior and Magnetic Resonance Imaging of Bladder Cancer

**DOI:** 10.1155/2021/1124526

**Published:** 2021-10-26

**Authors:** Hengxin Qi, Yuefeng Pan, Li Chen, Rui Li, Chonghua Wang, Ruimin Wang

**Affiliations:** ^1^Department of Imaging, Zhangqiu District People's Hospital, Jinan, China; ^2^Department of Imaging, People's Hospital of Rizhao, Rizhao, China; ^3^Operation Room, Zhangqiu District People's Hospital, Jinan, China; ^4^Department of Endocrinology, Zhangqiu District People's Hospital, Jinan, China; ^5^Department of Pediatrics, Zhangqiu District People's Hospital, Jinan, China

## Abstract

**Objective:**

This study aimed to investigate the effects of traditional Chinese medicine (TCM) on biological behavior and magnetic resonance imaging and recurrence rate of patients with bladder cancer.

**Method:**

Forty-seven postoperative bladder cancer patients treated in our hospital who met the criteria were selected and randomly divided into the TCM treatment group (observation group) and the group without TCM treatment (control group). In the TCM treatment group, the prescription was slightly adjusted according to the different symptoms, and the main prescription remained unchanged. According to the treatment plan, patients continued to undergo bladder irrigation chemotherapy plus TCM treatment, while the control group was only treated with bladder irrigation chemotherapy. The number of patients with recurrence at 3 and 6 months and 1 year, the effects on patients' clinical symptoms, and quality of life were observed, respectively. The changes in MRI images, blood routine, immune function, and leukocyte level and other related indexes before and after treatment were compared between the two groups.

**Results:**

After the patients in the observation group were treated with traditional Chinese medicine, the patients' quality of life significantly improved. The patients' CD3+, CD4+, and CD4+/CD8+ indexes were significantly higher than those of the control group. The levels of Hb and PLT of the patients in the observation group were significantly lower than those of the patients in the control group. Patients in the observation group had higher leukocyte levels and a lower recurrence rate than patients in the control group.

**Conclusion:**

TCM with chemotherapy drugs can effectively improve patients' immune function, increase the level of T-lymphocyte subpopulation, and improve bone marrow hematopoietic function, which has a significant effect on the prevention and treatment of bladder cancer recurrence after surgery.

## 1. Introduction

Bladder cancer is one of the most common malignant tumors of the genitourinary system, which seriously endangers human physical and mental health [1, 2]. Globally, bladder cancer is the ninth most prevalent malignant tumor, ranking sixth in men and about tenth in women [3–5]. Clinically, bladder cancer is often divided into nonmuscle invasive bladder cancer and muscle invasive bladder cancer. Nonmuscle invasive bladder cancer accounts for approximately 70%–75% of primary bladder tumors [6, 7], and it is generally less differentiated, more malignant, and more likely to develop into muscle invasive bladder cancer [8]. Bladder cancer often recurs, with its recurrence rate ranging from 20% to 70%, and up to 30% of patients eventually experience bladder cancer progression [8, 9]. And it is highly prone to recurrence after surgery, which has become a challenge for current clinical treatment [10–13].

Bladder cancer survival is approximately 16–20 months [14], and some patients with advanced bladder cancer do not achieve the expectation of controlling their disease after extensive radiotherapy and chemotherapy, and even aggravate their disease. The intervention of Chinese medicine can accelerate the recovery of patients, reduce the recurrence rate of surgery, improve the symptoms of side effects of surgery and perfusion therapy, and also play a more desirable consolidation role. TCM is a holistic approach to identifying and examining the causes of bladder cancer. It is believed that the pathogenesis of bladder cancer is mainly due to weakness of vital qi, and blood stasis, dampness, and heat toxicity are entangled with each other, resulting in a tangible mass over time. Pathogenesis based on root deficiency and branch excess: root deficiency presents with spleen-liver-kidney insufficiency and branch excess with phlegm and qi-blood stagnation. From the perspective of the four types of evidence, namely, dampness and heat, blood stasis and internal obstruction, spleen and kidney deficiency, and yin deficiency and internal heat, the dialectical use of Chinese medicine in the treatment of bladder cancer has achieved satisfactory outcomes.

Surgery, chemotherapy, and radiotherapy can play a certain role in bladder cancer, but not sufficient and high incidence of adverse reactions after the participation of radiotherapy and chemotherapy; it seriously reduces patients' quality of life and affects their confidence in actively accepting treatment, which in turn affects the desired outcomes. Therefore, in recent years, clinical practice has gradually strengthened the attempts to use Chinese medicine combined with Western medicine in the treatment of bladder cancer and has achieved better efficacy. The application of chemotherapy drugs is often accompanied by serious gastrointestinal reactions, bone marrow suppression, neurological damage, and other toxic side effects, and many patients often end their treatment midway because they have difficulty in tolerating the severe side effects of chemotherapy. In the treatment of bladder cancer, the application of bladder irrigation with Chinese medicine tonics has an inhibitory effect on white corpuscle.

With the continuous development and improvement of medical technology, diagnostic imaging technology has been widely used. At present, imaging technology has become an essential method for diagnosing bladder cancer. In clinical experiments, the application of imaging technology can be used to identify patients' bladder cancer lesions, so that medical personnel can better understand patients' physical conditions and thus adopt suitable treatment plans, so that bladder cancer patients can receive timely and effective treatment. There are two types of magnetic resonance imaging, diffusion-weighted imaging, and MR elastography. Diffusion-weighted imaging is an imaging technique obtained by the difference in the motion of water molecules between tissues. The problems concerning motion have been overcome by the application of MRI, which is mainly used to examine the imaging data of the abdomen. Diffusion-weighted imaging does not involve other contrast agents and the acquisition time is relatively short compared to ultrasound diagnosis. In clinical trials, MRI diffusion-weighted imaging is mainly used for imaging detection of bladder cancer tumors. In addition, it can make effective detection of bladder cancer lesions, so that the corresponding treatment plan can be formulated for the histological grading of bladder cancer, and the recurrence of bladder cancer can be prevented.

MRI scans have wide use nowadays. In recent years, with the continuous development of hardware and software, functional magnetic resonance imaging (fMRI) has been gradually applied to the study of abdominal organs and lesions. In this study, we selected “bladder cancer patients” as the study objects and initially investigated the effect of Chinese medicine on the recurrence of bladder cancer after surgery, as well as the improvement of clinical symptoms and quality of life. As an important supplement to conventional MRI scanning, functional magnetic resonance imaging has now become a popular research and application direction.

## 2. Materials and Methods

### 2.1. Research Objects

47 patients at the Oncology and Gynecology Departments of Zhangqiu District People's Hospital, Jinan, Shandong, China, between January 1, 2020, and May 31, 2021, were included in this study, and all patients had complete clinical data. Among them, there were 35 male patients and 12 female patients, aged 35–80 years, with a mean age of 58.2 years. There were 5 cases at clinical stage T0, 31 cases at stage T1, and 11 cases at stage T2. There were 15 cases of pathological grade I and 32 cases of grade II, all of which underwent resection of bladder tumor with pathological diagnosis reports. There were 29 cases of noninvasive bladder cancer and 18 cases of invasive bladder cancer. All patients were treated with TURBT surgery and bladder perfusion chemotherapy. The patients were divided into the TCM treatment group (observation group, 24 cases) and the group without TCM treatment (control group, 23 cases). Some patients were found to have recurrence after treatment, and the number of recurrences ranged from 2 to above 30. This study was approved by the ethics committee of Zhangqiu District People's Hospital, Jinan, Shandong, China, and all patients gave informed consent.

### 2.2. Inclusion Criteria

1. Patients who had been diagnosed with bladder cancer, had pathological diagnoses, and underwent surgery.
2. Patients between the ages of 35 and 70 years.
3. Patients who voluntarily participated in the study and had signed the informed consent form.
4. Performance status (KPS) score >60 and expected survival >12 months.
5. Patients with no psychiatric or psychiatric history that would affect informed consent and who had some communication and language skills.
6. Patients with no other malignancies and severe comorbidities.
7. Patients with complete medical information.

### 2.3. Exclusion Criteria

1. Patients with significant preoperative inflammatory reactions, combined with severe primary diseases of the heart, liver, kidney, blood or endocrine system, and psychiatric and immune disorders
2. Patients who had not undergone postoperative bladder irrigation or who had not been treated with formal irrigation.
3. Patients who had other malignant systemic diseases.
4. Patients with a perioperative application of antibiotics, long-term use of drugs that suppressed the immune system, and hormonal drugs.
5. Poor patient compliance and reluctance to accept surveys.
6. Patients lost to follow-up.

### 2.4. General Information

The patient's clinical information mainly covered basic personal information, history, blood test results about one week before surgery, surgical records, pathology reports, and so on. Basic personal information includes the patient's age, gender, contact information (for follow-up), and blood results about one week before surgery. History includes a history of smoking and a history of diseases. Contents of surgical records include tumor size and number, tumor shape, and location. Pathology report includes the degree of pathological differentiation and whether it is infiltrating muscle layer (Table 1).

### 2.5. Treatment Method

The basic formula of Chinese medicine was as follows: glabrous greenbrier rhizome, Yuge, chrysanthemum flower, prepared rehmannia root, villous amomum fruit, asiatic cornelian cherry fruit, common yam rhizome, tree peony root bark, oriental water plantain rhizome, milkvetch root, cassia bark, common selfheal fruit-spike, and gecko.

The above herbs were taken by decoction with water twice a day, 1 dose/day, for at least six months. The patients did not eat cold and greasy food during the medication period, with recording the change of symptoms and followed up every two weeks at the outpatient clinic.

Bladder irrigation is routine intravesical chemotherapy drug and immunosuppressant irrigation therapy.

### 2.6. Observation Time and Follow-Up

From the 1^st^ dose of Chinese medicine, follow-up was conducted by regular outpatient review and telephone follow-up.

  Review time: patients were reviewed once every 3 months in the first year after surgery and once every 6 months from the second year onwards.
  Review items: physical examination, MRI-based imaging, abdominal CT or ultrasound and cystoscopy, etc., combined with cystoscopy biopsy for pathology if necessary, and the number of patients with recurrence was derived from the collected follow-up data.

### 2.7. Observation Contents

#### 2.7.1. Tumor Recurrence

The patient was treated with transurethral bladder tumor electrosurgery and returned to the hospital for follow-up urological CT and cystoscopy in the 3^rd^, 6^th^, and 12^th^ months after surgery to observe the postoperative recurrence.

#### 2.7.2. Adverse Drug Reactions

Patients were observed to receive bladder irrigation chemotherapy followed by treatment with Chinese medicine for drug side effects, including symptoms such as carnal hematuria, urinary frequency, urinary urgency, urinary pain, and lower abdominal pain.

#### 2.7.3. Changes in Immune Function

Before and after the treatment, 5 mL of fasting venous blood was taken from the patients and placed on our automatic blood centrifuge for centrifugation, the speed of the centrifuge was adjusted to 3000 r/min for 10 min, and the supernatant was placed in a refrigerator at −20 for examination. The T-lymphocyte subsets in the serum were detected.

#### 2.7.4. Blood Routine Examination

Before and after the treatment, 5 mL of fasting venous blood was taken from the patients and placed on our automatic blood centrifuge for centrifugation, the speed of the centrifuge was adjusted to 3000 r/min for 10 min, and the supernatant was placed in a refrigerator at −20 for examination. The hemoglobin (Hb) and platelet (PLT) count of the patients was tested before and after the treatment.

#### 2.7.5. Leukocyte Level

The efficacy was evaluated according to the grading criteria for myelosuppression by chemotherapy: degree I, 3.0 × 10^9^/*L* ≤ WBC<4.0 × 10^9^/L; II, 2.0 × 10^9^/*L* ≤ WBC<3.0 × 10^9^/L; III, 1.0 × 10^9^/*L* ≤ WBC<2.0 × 10^9^/L; and IV, WBC<1.0 × 10^9^/L.

#### 2.7.6. Magnetic Resonance Imaging

The patient was put in the supine position with a proper bladder filling by fasting for 6 h before the examination with a 1.5 T (MAGNETOM Avanto) scanner. The parameters were set as follows: HR-T2WI (TR of 7000–8 000 ms, TE of 90–102 ms, layer thickness of 3 mm, layer spacing of 1 mm); DWI (TR of 4 000 ms, TE of 78 ms, layer thickness of 4 mm, layer spacing of 0.4 mm); and DCE (TR of 180–300 ms, TE of 1.7–4, layer thickness of 6 mm, layer spacing of 2 mm, reversal angle 70°). The patient was injected with Magenvixen through the elbow vein at a uniform rate, the multiphase dynamic enhancement images were obtained at 20, 30, 40, 60, 80, and 100 s after the injection, and the delayed phase scan was performed 3 min later. The MRI was performed by two senior physicians in the imaging department of our hospital.

### 2.8. Statistical Analysis

SPSS 22.0 software was applied to process and analyze the data in this study, and the measurement data were described by mean ± standard deviation ($\bar{x}\;\pm \;s$). A *t*-test was used for comparison, the count data were described by rate or percentage (%), and the chi-square test was used for comparative analysis. *P* < 0.05 was a statistically significant difference.

## 3. Results

### 3.1. Recurrence of Bladder Cancer One Year after Surgery

The number of recurrences within 3 months was 2 cases, both in the control group (8.7%), and there was no recurrence in the observation group (Table 2). The recurrence rate in the control group was 13.0% within 6 months, and the recurrence rate in the observation group was 4.2%, which was significantly lower than the recurrence rate in the control group. Seven cases recurred within 12 months: two in the observation group, with a recurrence rate of 8.3%, and five in the control group, with a recurrence rate of 21.7%. This indicated that the combined treatment of Chinese and Western medicine was effective in preventing the recurrence of bladder cancer after surgery.

### 3.2. MRI of Patients after Chinese Medicine Treatment

Postoperative MRI showed that T1WI signal was increased to different degrees, 3 of which had uniform high signal, 1 had uniform isointensity signal, and the rest had mixed signal. For T2WI, 1 had uniform high signal, 4 had uniform low signal, and 1 had uniform isointensity signal. DWI showed that 9 lesions had high signal, and the rest had varying degrees of signal decrease. Dynamic enhancement scans showed no significant arterial phase enhancement within any of the 25 treated areas, one marginal arterial phase enhancement, and seven delayed scans showed mild marginal enhancement (Figure 1). The pathological picture of 400 times a different installment of bladder cancer is shown in Figure 2.

MRI image of patient A showed a small amount of cancer involvement in the smooth muscle and fibrous connective tissue (of the bladder tumor base) and the pathological diagnosis indicated that patient A was high-grade invasive uroepithelial carcinoma with a small percentage of micropapillary carcinoma (about 2%) (Figure 1A). The MRI image of patient B is shown in Figure 1B. The pathologic diagnosis showed mucosal ulcer formation in the right side of the bladder wall within the total cystectomy specimen, reaching deep into the muscular layer, with interstitial edema and necrosis with more chronic inflammatory cell infiltration. After adequate sampling (11 wax blocks), no cancer residue was seen, and no cancer involvement was seen in the prostate and bilateral seminal vesicle glands and vas deferens. No metastasis was observed in the left pelvic (0/5) and right pelvic (0/1) lymph nodes.

MRI image of patient C (Figure 1C) showed bladder tissue, prostate, and bilateral vesicoureteral glands and vas deferens. The bladder size was 5*∗*4*∗*4.5 cm, and a rough mucosal area (3*∗*2 cm) was seen on the right side, which seemed to invade the muscle layer. The prostate size was 3.5*∗*3.5*∗*2.7 cm. The size of the left seminal vesicle gland was 2.4*∗*1.5*∗*0.7 cm, the length of the left vas deferens was 7 cm and the maximum diameter was 0.5 cm, the size of the right seminal vesicle gland was 3.2*∗*2*∗*0.7 cm, and the length of the right vas deferens was 7.5 cm and the maximum diameter was 0.7 cm. The left pelvic lymph nodes were covered with grayish-yellow fatty tissue with a combined size of 4.5*∗*3*∗*1.5 cm and several enlarged lymph nodes with a maximum diameter of 1–1.7 cm. The right pelvic lymph nodes were covered with one grayish-yellow fatty tissue and one enlarged lymph node with a maximum diameter of 2 cm. Combined with pathological diagnosis, this patient was diagnosed with high-grade uroepithelial carcinoma (microscopic diameter of approximately 0.3 cm) with squamous. The invasion reached the lamina propria and did not involve the urethral margin, prostate, bilateral seminal vesicle glands, and vas deferens. No metastasis was found in the lymph nodes of the left pelvis (0/6) and right pelvis (0/3).

### 3.3. Adverse Reactions to Bladder Irrigation Drugs

Adverse reactions during treatment were recorded and evaluated in 47 patients in both groups using the Common Terminology Criteria for Adverse Reactions, version 5.0. Two patients in the observation group were recorded with malaise, one with hypothermia, and zero with weight loss after treatment, while five patients in the control group were recorded with malaise, three with hypothermia, and one with weight loss after treatment. In the control group, 2 patients showed mild gastrointestinal reactions with decreased appetite and no vomiting symptoms, and 1 patient showed constipation during treatment. In the observation group, there were 8 cases of gastrointestinal reactions. 11 patients in both groups had symptoms such as urinary frequency, urinary urgency, urinary pain, hematuria, and lower abdominal pain, the incidence of which was 12.5% in the observation group and 34.8% in the control group. None of the 47 patients experienced toxic reactions other than gastrointestinal symptoms and systemic symptoms, and no urethral strictures occurred (Table 3). The results showed that Chinese medicine did not aggravate or persist in adverse reactions and significantly reduced the incidence of adverse reactions in patients after bladder irrigation chemotherapy.

### 3.4. Leukocyte Levels

The recurrence rate of bladder cancer after surgery is high, so the method of camptothecin bladder infusion is mainly used after surgery to prevent its postoperative recurrence or metastasis. The application of chemotherapeutic drugs is often accompanied by severe gastrointestinal reactions, bone marrow suppression, nerve damage, and other toxic side effects. Many patients often end their treatment midway because they have difficulty tolerating the toxic side effects of chemotherapy. However, the bone marrow suppression of camptothecin local chemotherapy is mostly the suppression of leukocytes, so the application of Chinese medicine treatment to improve the suppression of leukocytes by camptothecin is of great clinical significance. After the application of traditional Chinese medicine in this study, it could be seen from Figure 3 that the leukocyte level in the control group was 3.21 ± 1.24, and after traditional Chinese medicine treatment, the leukocyte level was 4.37 ± 1.23, and there was a significant difference in the leukocyte count between the two groups (*P* < 0.05). Results showed that the leukocyte count after traditional Chinese medicine treatment was significantly higher than that of the patients in the control group, suggesting that traditional Chinese medicine could effectively enhance the body's immune and the bone marrow hematopoietic capacity of bladder cancer patients after surgery.

### 3.5. Comparison of Indicators Related to T-Lymphocyte Subsets

Although radiotherapy and chemotherapy for bladder cancer after surgery can prolong patients' disease-free survival and reduce mortality, most patients have apparent adverse effects and suppressed immune function. Immunological studies have shown that the occurrence, development, and prognosis of tumors are directly related to the immune function of the body, especially the T cell-mediated cellular immunity. T cells mainly include two subpopulations: CD4+ and CD8+. Traditionally, CD4+ is considered as helper T cells and CD8+ as suppressor T cells, so the ratio of CD4+, CD8+, and CD4+/CD8+ cells is measured to directly reflect the cellular immune function of patients.

The level of CD3+ was 53.12 ± 6.24 in the control group and 60.23 ± 7.14 in the observation group, and the level of CD3+ was elevated by Chinese medicine treatment. The CD4+ in the control group was 40.21 ± 5.12 and 49.01 ± 3.48 in the observation group. The CD8+ and CD4+/CD8+ in the control group were 35.23 ± 4.87 and 1.14 ± 0.17 and 31.68 ± 3.92 and 1.55 ± 0.16 in the observation group, respectively. The results showed that the levels of CD3+ and CD4+ were significantly increased, the CD8+ level was decreased, and CD4+/CD8+ was significantly increased compared with the control group (*P* < 0.05), suggesting that the use of traditional Chinese medicine can effectively enhance the immune function of the body of bladder cancer patients after surgery (Figure 4).

### 3.6. Comparison of Blood Routine Related Indexes between Two Groups of Patients before and after Treatment

The platelet, neutrophil, and hemoglobin levels of patients with bladder cancer after surgery were normal, indicating that traditional Chinese medicine did not cause abnormal changes in blood routine and adverse reactions. In addition, the application of traditional Chinese medicine could effectively reduce the side effects produced by chemotherapy. The Hb and PLT levels of patients in the control group were 121.33 ± 12.32 g/L and 209.31 ± 11.97 109/L, respectively, and the Hb and PLT levels of the observation group were 102.34 ± 6.14 g/L and 161.21 ± 9.74 109/L, respectively. After treatment with traditional Chinese medicine, the Hb and PLT levels were significantly lower in the control group than the observation group (*P* < 0.05, Figure 5).

### 3.7. Improvement in Quality of Life

Patients' symptom improvement and quality of life were scored from the first day of treatment to the end, with reference to the clinical symptom score (Figure 6) and Carlsbad score (Figure 7) in both groups. The clinical symptom scores of patients in the observation group were (21.32 ± 3.01) significantly increased compared to the patients in the control group (8.72 ± 2.87), which illustrated that Chinese medicine could improve the quality of life of patients (Figure 6).

## 4. Discussion

Bladder cancer is one of the most common urinary system cancers and is receiving increasing attention because of its high incidence and recurrence rate. Moreover, due to the improvement of living standards and related auxiliary examinations such as urological CT and cystoscopy, bladder tumors have been diagnosed earlier and more sensitively. NMIBC is preferred to be treated with TURBT, and MIBC is mostly treated with radical cystectomy or bladder-preserving combination therapy.

Recurrence occurs in 60% to 70% of NMIBC patients within 1 to 2 years after TURBT treatment, and tumor recurrence may be at risk for higher malignancy and greater invasive and metastatic capabilities [15]. The occurrence of bladder cancer is multicentric, and the possibility of cancer cell shedding and implantation inevitably exists preoperatively and intraoperatively. The possibility of incomplete tumor removal exists in both TURBT and partial cystectomy, which may be partly responsible for the recurrence and progression of bladder tumors. Moreover, the higher recurrence rate and possible accompanying tumor progression are important reasons affecting their prognosis. Therefore, to improve the prognosis of bladder cancer, complete removal of the tumor and the shed and grown cancer cells become the main purpose.

A safe, noninvasive, and relatively accurate way of preoperative diagnosis, postoperative outcome assessment, and prediction is sought to improve long-term survival. CT and MRI are now commonly used for imaging to evaluate efficacy. However, CT has limitations due to radiation and false negatives and difficulty in characterizing some recurrent lesions. In contrast, MRI is free of radiation concerns and has a high soft-tissue resolution. MRI provides more diagnostic information and facilitates the detection of residual or recurrent lesions. Magnetic resonance diffusion-weighted imaging (MRI-DWI) is a noninvasive imaging technique that belongs to functional imaging. It reflects the information of living tissue structure and cell density by detecting the diffusion motion of water molecules. It is the only method to observe the movement of water molecules in the body and has been maturely applied to imaging neurological diseases.

The results of this study showed that the percentage of CD4+ and CD3+ cells and the CD4+/CD8+ ratio of patients in the observation group were significantly increased compared with the control group (*P* < 0.05). Better clinical results were achieved, and no adverse effects were observed throughout the drug administration. Our findings suggest that the use of traditional Chinese medicine treatment could significantly improve the cellular immune function of the body, improve the hematopoietic function of bone marrow, and have fewer toxic side effects, which has a certain effect on the prevention of recurrence and metastasis after bladder cancer surgery. For postoperative residual or recurrent lesions, through long-term follow-up review and MRI-DWI image control analysis, most of the residual or recurrent tumors were located in the marginal part of the original cancer foci; the appearance of slightly longer signals at the margins after TURBT often suggested recurrence; dynamic enhancement scans showed fast-in and fast-out performance; the scope of recurrent lesions would increase with longer follow-up time; and the time of recurrence was mainly 12 months after surgery. Long-term follow-up review and MRI-DWI image control analysis revealed that most of the tumor residuals or recurrences were located in the marginal part of the original cancer foci. The appearance of slightly longer signals at the margins after TURBT often suggested recurrence; dynamic enhancement scans showed fast-in and fast-out manifestations; the scope of recurrent lesions increased with longer follow-up time; and the recurrence time was mainly 12 months after surgery. However, the number of cases in this study was small and the observation and follow-up period was short. In addition to the continued follow-up of existing cases, a larger, multicenter, prospective, and longer-term clinical study was needed to confirm the value of the application of Xiaoji Shenqi Decoction.

## 5. Conclusion

The efficacy of Chinese medicine in preventing the recurrence of bladder cancer after surgery was satisfactory, and it had a higher recurrence-free survival with a higher safety profile. Hence, it merits encouragement in clinical application.

## Figures and Tables

**Figure 1:** MRI image of the patient. Uppercase letters represented the patient's preoperative images and lowercase letters represented the patient's postoperative images.

**Figure 2:** Pathological pictures of different stages of bladder cancer (×400). (a) T0. (b) T1. (c) T2.

**Figure 3:** Comparison of leukocyte levels between the observation group and the control group. ^*∗*^*P* < 0.05.

**Figure 4:** Comparison of indicators related to T-lymphocyte subsets in two groups of patients. ^*∗*^*P* < 0.05.

**Figure 5:** Comparison of routine blood-related indicators between two groups of patients. ^*∗*^*P* < 0.05.

**Figure 6:** Clinical symptom score of each clinical symptom between two groups of patients. ^*∗*^*P* < 0.05; ^*∗∗*^*P* < 0.01.

**Figure 7:** Carlsbad score of patients in both groups. ^*∗*^*P* < 0.05.

**Table 1:** General characteristics of the patients.

Characteristics		Observation group (24 cases)	Control group (23 cases)
Gender	Male	17 (70.8%)	18 (78.3%)
	Female	7 (29.2%)	5 (21.7%)
Age		59.2 ± 5.01	57.3 ± 6.24
Number of tumors	Single	7 (29.2%)	8 (34.8%)
	Multiple	17 (29.2%)	15 (5.2%)
Maximum tumor diameter		37.21	36.67
Clinical stage	T0	2 (8.3%)	3 (13.0%)
	T1	16 (66.7%)	15 (65.2%)
	T2	6 (25.0%)	5 (21.7%)

**Table 2:** Bladder cancer recurrence rate.

Time	Group	Cases	Recurrence	No. of recurrence	Recurrence rate (%)
3 months	Observation group	24	0	24	0
	Control group	23	2	21	8.7
6 months	Observation group	24	1	23	4.2
	Control group	23	3	20	13.0
12 months	Observation group	24	2	22	8.3
	Control group	23	5	18	21.7

**Table 3:** Incidence of adverse reactions to bladder irrigation chemotherapy.

Characteristics		Observation group	Control group
Systemic symptoms	Malaise	2 (8.3%)	5 (21.%)
	Hypothermia	1 (4.2%)	3 (13.0%)
	Weight loss	0	1 (4.3%)
Skin reaction		0	1 (4.3%)
Gastrointestinal reactions	Vomiting	0	1 (4.3%)
	Anorexia	1 (4.2%)	3 (13.0%)
	Constipation	1 (4.2%)	4 (17.4%)
Other adverse reactions	Frequent urination	3 (12.5%)	8 (34.8%)
	Urinary urgency		
	Painful urination		
	Lower abdominal pain		

## Data Availability

The data used to support the findings of this study are available from the corresponding author upon request.
